# GABPA Expression in Endometrial Carcinoma: A Prognostic Marker

**DOI:** 10.1155/2021/5552614

**Published:** 2021-06-29

**Authors:** Xiaoxue Ma, Qianhan Lin, Gongting Cui, Jing Zhao, Xuan Wei, Rui Li, Hongluan Mao, Yanhui Ma, Peishu Liu, Yingxin Pang

**Affiliations:** ^1^Department of Obstetrics and Gynecology, Qilu Hospital of Shandong University, Jinan 250012, China; ^2^Key Laboratory of Gynecology Oncology of Shandong Province, Qilu Hospital, Jinan 250012, China; ^3^Department of Pathology, People's Hospital of JiaXiang, Jining 272400, China; ^4^Shandong Engineering Laboratory for Urogynecology, Jinan 250012, China

## Abstract

**Background:**

GA-binding protein A (GABPA), a transcription factor, is broadly involved in physiological and pathological processes. Several studies have investigated the relationship between GABPA expression level and outcomes of various malignancies. However, the function and clinicopathological significance of GABPA in endometrial carcinoma (EC) remain obscure.

**Methods:**

The GABPA mRNA expression in EC tissues and adjacent nonneoplastic tissues in the TCGA database was involved in our study. The protein expression of GABPA in 107 EC tissues and 15 normal endometrial tissues was detected by immunohistochemistry.

**Results:**

The GABPA expression was significantly downregulated in EC tissues compared with its expression in normal tissues (*P* < 0.001). The expression of GABPA was markedly correlated with type II EC (*P* < 0.01) and grade 3 EC (*P* < 0.05). A tendency has been observed that patients with low GABPA levels had relatively poorer overall survival (OS) (*P* = 0.036) and disease-free survival (DFS) (*P* = 0.016) than patients with high GABPA levels. The multivariate Cox proportional hazard model showed that lower expression of GABPA was an independent poor prognostic factor for OS (*P* = 0.043) and DFS (*P* = 0.045). Similar correlation between low expression levels of GABPA and unfavorable prognosis has also been found in type II or grade 3 EC. IHC analysis showed EC tissues had low expression of GABPA, which indicated relatively poor prognosis. Moreover, we identified that the GABPA mRNA expression was negatively correlated with its methylation level (*R* = −0.2512, *P* < 0.001) which is one of the mechanisms for the silencing of GABPA gene.

**Conclusion:**

GABPA may act as an independent predictor of clinical prognosis and serve as a potential target gene for EC therapy.

## 1. Introduction

Endometrial carcinoma (EC) is one of the most common gynecologic malignancies with a rising incidence by approximately 1.3% per year over the last 10 years. It is estimated that about 65,620 new EC cases will be diagnosed in the United States and around 12,590 women will die from EC in 2020 [1]. It mainly occurs in women between 55 and 65 years old [2]. But with the continued declines in the fertility rate and the increased obesity, the incidence of EC is on the rise in young women [1]. Current EC treatment strategies include surgery and adjuvant therapy, such as chemotherapy, radiotherapy, hormonal therapy, and immunotherapy. Surgery is the first-line treatment for EC, which is also the basis for comprehensive treatment of the disease, especially for early-stage EC. High-risk EC is characterized by higher grades, advanced stages, or nonendometrioid histology [3]. About 15% to 20% of patients with EC present with high-risk disease and have poorer prognosis [4]. Despite new antitumor agents and more effective combination treatments, it has been reported that the 5-year survival rate of stage IV patients is approximately 17% [5]. Therefore, it is important to explore new molecular markers and identify potential therapeutic targets.

The E26 transformation-specific (ETS) family of transcription factors comprises 30 different members, which plays critical roles in development, cell differentiation, and oncogenesis [6]. GA-binding protein A (GABPA) is unique among the ETS factors, which is an obligate multimeric protein complex regulating DNA binding and transcription [7]. In addition, GABPA interacts with other transcription factors or coactivators to regulate the expression of various genes which participate in a series of complex physiological and pathological processes [8].

GABPA is involved in the maintenance and differentiation of hematopoietic stem cells (HSCs) by activating the transcription of DNA methyltransferases and histone acetylases [9]. In addition, GABPA is required for proliferation and differentiation of both myeloid and lymphoid cells [10, 11]. GABPA also controls the expression of genes involved in the mitochondrial function, and its inactivation results in early embryonic lethality [12]. Additionally, GABPA plays a major direct role in cell cycle progression [13, 14]. It was previously reported that conditional deletion of GABPA in mouse embryonic fibroblasts (MEFs) leads to dysfunction in cell cycle progression, including delay in G1 to S transition and reduce in the numbers of cells entering the cell cycle [15, 16]. Several studies have revealed that the abnormal expression of GABPA was related to poor survival in various cancers, including leukemia, hepatocellular carcinoma, thyroid cancer, bladder cancer, and prostate cancer [6, 17–22]. The involvement of GABPA in EC remains unclear.

In order to assess whether GABPA may serve as a prognostic factor for EC, we examined the GABPA expression in mRNA and protein levels in EC tissues. And the relationship between the expression levels of GABPA and clinicopathological characteristics and its prognosis value in EC was evaluated. Moreover, we have initially explored the mechanism on the downregulation of the GABPA expression.

## 2. Materials and Methods

### 2.1. TCGA Datasets

The Cancer Genome Atlas (TCGA) project, which was launched by the National Cancer Institute and the National Human Genome Research Institute, is a landmark program aiming to comprehensively elucidate molecular changes during carcinogenesis and tumor progression and to link cancer genomic data to patients' clinical information. The RNA-seq expression data (543 cases), clinical data, and methylation data (as detected by Illumina HumanMethylation450 BeadChip) were downloaded from TCGA official website for the Uterine Corpus Endometrial Carcinoma (UCEC) project in October 2019.

### 2.2. Patients and Specimens

From February 2010 to December 2014, 107 EC tissues and 15 nonmalignant tissues were selected from the Department of Pathology of Qilu Hospital of Shandong University for paraffin section. None of the patients received chemotherapy or radiotherapy before the operation. Our study was approved by Medical Ethics Committee of Qilu Hospital of Shandong University. All samples were deidentified and provided as completely anonymous samples. Follow-up data of all patients were obtained by interview or telephone.

### 2.3. Hematoxylin-Eosin and Immunohistochemistry Staining

Tissues were fixed with 10% neutral formalin and embedded in paraffin, and 4 *μ*m-thick sections were prepared by the pathology technologist. For hematoxylin-eosin staining (H&E) staining, sections were dewaxed and hydrated with a gradient of alcohols. After immersion in phosphate buffered saline (PBS), the sections were stained with H&E. Immunohistochemistry (IHC) staining was performed by standard staining procedures as described previously [23]. GABPA antibody (1 : 50, 21542-1-AP) was purchased from Proteintech (Wuhan, China).

### 2.4. Evaluation of Immunostaining

The expression of GABPA was assessed according to the immunoreactive score (IRS), determined by evaluating the proportion of positive tumor cells, scored as 0 (≤5% positive tumor cells), 1 (6-25% positive tumor cells), 2 (26-50% positive tumor cells), 3 (51-75% positive tumor cells), and 4 (≥76% positive tumor cells) and the intensity of their staining, graded as 0 (negative), 1 (weak), 2 (moderate), and 3 (strong). The staining intensity score was then multiplied by the proportion of positive cells to obtain the immunoreactive score for each sample, ranging from 0 to 12. In order to facilitate statistical evaluation, the GABPA protein expression level was reclassified according to semiquantitative scheme. Low levels of expression were defined as immunoreactive score < 6, and high levels of expression were defined as immunoreactive score ≥ 6.

### 2.5. Statistical Analysis

Statistical analysis is performed using GraphPad Prism 8.0 (GraphPad Software, San Diego, CA, USA) and IBM SPSS 21.0 software (IBM SPSS, Armonk, NY, USA). Detailed statistical methods were described previously [23]. The relationship between GABPA gene methylation level and mRNA expression was explored by correlation analysis. Statistical significance was determined by*P* < 0.05.

## 3. Results

### 3.1. Expression of GABPA mRNA and Clinicopathological Characteristics in EC Patients

RNA-seq and clinical data of 543 patients suffered EC were downloaded from the TCGA official website for the UCEC. No patient had a history of neoadjuvant therapy. Patients with a previous cancer history or multiple primary neoplasms at the time of diagnosis, patients whose follow-up time was less than 30 days or over 8 years after surgery, and patients who recurred or died within 30 days after operation were excluded. Finally, 490 patients in TCGA were involved in analysis. In order to define the true “high level” and “low level,” the patients carrying EC from TCGA were divided into two groups, expressing either low (*n* = 245) or high GABPA levels (*n* = 245) (Table 1).

The clinicopathological characteristics of 490 patients carrying EC involved are summarized in Table 1. Patients' mean age was 63.70 (standard deviation = 11.87), and most patients were with stage I EC (62.86%). Majority of patients (76.94%) were diagnosed with endometrioid endometrial adenocarcinoma, followed by serous endometrial adenocarcinoma (18.78%) and mixed type (4.28%). In all, patients carrying grade 3 EC (58.16%) are most common. Other clinical characteristics are detailed in Table 1.

The GABPA expression was significantly downregulated in EC tissues compared with its expression in normal endometrium tissues (*P* < 0.001) (Figure 1(a)). Consistent with this finding, analysis in 23 paired samples showed that the GABPA expression was significantly lower in EC than in adjacent normal tissues (*P* < 0.001) (Figure 1(b)), and the GABPA expression in EC of all pathological types decreased significantly compared with normal endometrium tissues (*P* < 0.001) (Figure 1(c)). Moreover, GABPA expression was significantly related to type II EC (*P* < 0.01) (Figure 1(d)) and grade 3 EC (*P* < 0.05) (Figure 1(e)). However, there is no significant correlation between GABPA expression and tumor stage (*P* > 0.05) (Figure 1(f)).

### 3.2. GABPA mRNA Expression and Survival Time Analysis in EC Patients

Kaplan-Meier survival analysis was used to evaluate the prognostic value of GABPA in EC patients. Patients with low expression levels of GABPA had relatively poorer OS than patients with high expression levels of GABPA (HR: 0.488, CI: 0.258-0.922, *P* = 0.036) (Figure 2(a)). We also found the similar tendency in DFS (HR: 0.585, CI: 0.381-0.897, *P* = 0.016) (Figure 2(b)).

Given that type II EC is associated with poor prognosis, we further analyze the expression of GABPA in type II EC patients. Compared with the low expression group, the high expression group exhibited better OS (HR: 0.290, CI: 0.096-0.874, *P* = 0.016) and DFS (HR: 0.406, CI: 0.182-0.905, *P* = 0.018) in type II EC (Figures 3(a) and 3(b)). In addition, we found that the low expression of GABPA was negatively correlated with OS (HR: 0.383, CI: 0.187-0.784, *P* = 0.012) in patients with grade 3 EC, and the similar findings were also presented in the analysis of DFS (HR: 0.434, CI: 0.256-0.734, *P* = 0.002) (Figures 3(c) and 3(d)).

### 3.3. Prognostic Value of GABPA mRNA in EC Patients

In univariate analysis, the low expression of GABPA was corresponded to poor prognosis of both OS (HR: 0.487, CI: 0.246-0.966, *P* = 0.040) (Table 2) and DFS (HR: 0.584, CI: 0.375-0.910, *P* = 0.018) (Table 3) in EC. Other clinicopathological characteristics associated with poor survival included type II, high grade, and advanced stage (Tables 2 and 3). In multivariate COX regression, GABPA was confirmed as an independent prognostic marker for OS (HR: 0.491, CI: 0.246-0.977, *P* = 0.043) (Table 2) and DFS (HR: 0.619, CI: 0.397-0.966, *P* = 0.045) (Table 3).

### 3.4. The Expression of GABPA Protein and Clinicopathological Characteristics in EC Patients

In order to further clarify the protein expression level and localization of GABPA in EC tissues, we performed IHC staining in a total of 107 EC tissues and 15 normal endometrium tissues. Follow-up data were available in 100 of 107 EC patients in the present cohort. The clinicopathological characteristics of EC patients were detailed in Table 4. The findings are in line with results from previous studies that patients with grade 1 tumors are the most common (43.93%), and those with grade 3 tumors are the least common (22.43%). Deep myometrial invasion was observed in 33.64% patients and cervical invasion in 9.35% patients. IHC staining revealed that the GABPA expression was highly heterogeneous among ECs (Figure 4) and distributed in both nucleus and cytoplasm. In this study, the IRS was based on nuclear staining because no significant correlations were found between the cytoplasmic staining and either the clinicopathological features or prognosis. The expression of GABPA in EC tissues was also decreased compared to normal tissues (Figure 5(c)). It also revealed that the low GABPA expression was seen in 59.81% (64/107) of EC patients.

### 3.5. The Expression of GABPA Protein and Prognosis in EC Patients

Next, the relationship of GABPA protein expression with OS in EC patients was assessed by Kaplan-Meier analysis and log-rank test. EC patients with the low GABPA expression had significantly shorter OS compared with those with high expression (HR: 0.257, CI: 0.103-0.638, *P* = 0.020) (Figure 6(a)). And we found the same trend in DFS (HR: 0.373, CI: 0.163-0.852, *P* = 0.042) (Figure 6(b)). These results suggested that patients with low GABPA expression had poorer prognosis. In multivariate COX regression, GABPA was confirmed as an independent prognostic marker for OS (HR: 0.267, CI: 0.078-0.918, *P* = 0.036) (Table 5).

### 3.6. Effects of DNA Methylation Level on the GABPA Expression

Finally, we sought to probe the mechanism of GABPA downregulation in cancers. The above observations indicate that GABPA may exhibit tumor suppressive function in EC. Aberrant promoter methylation is the predominant mechanism for silencing tumor suppressor genes. To determine whether the methylation of GABPA results in its suppression, we analyzed the relationship between the gene methylation level and mRNA expression of GABPA in ECs using TCGA. The results demonstrate that GABPA mRNA expression is negatively correlated with its gene methylation level (*R* = −0.2512, *P* < 0.001) (Figure 7(a)). Moreover, we identified one methylated CpG at cg21890848 of GABPA gene played a predominant role in its silence (*R* = −0.2506, *P* < 0.001) (Figure 7(b)). Above results indicated that aberrant methylation is one of the major mechanisms for the silencing of the GABPA gene.

## 4. Discussion

In present study, we found that the mRNA expression of GABPA was decreased in EC patients and correlated with EC prognosis using a bioinformatic analysis approach. Moreover, our study showed that the protein expression of GABPA was downregulated in EC tissues compared with normal endometrial tissues. Lower expression of GABPA was correlated with relatively poor prognosis. These data suggested that GABPA serves as a tumor suppressor in EC development and survival.

GABPA, a transcription factor, regulates the genes expression involved in various physiological and pathological processes, such as the embryonic development, mitochondrial function, innate and acquired immunity, cell cycle progression, and cell invasion and metastasis [12, 24]. Recent studies implied a complicated relationship between GABPA and tumor progression. Guo et al. indicated that GABPA dictates luminal identity of bladder cancer (BC) cells and inhibits aggressive diseases in BC by promoting cellular differentiation despite its stimulatory effect on telomerase/TERT activation [17]. Yuan and Paulsson et al. suggested that GABPA acts as a tumor suppressor by directly regulating DICER1 in follicular and papillary thyroid tumors [19, 22]. Zhang et al. indicated that GABPA inhibits HCC cell migration by modulating E-cadherin and acts as a tumor suppressor [18]. However, the current mechanisms of GABPA on cancer initiation and progression are inconsistent. A study showed that GABPA plays as a complex role in controlling breast epithelial cell migration by directly affecting the expression of RAC2 and KIF20A [25]. Sharma et al. found that GABPA mediates malignant phenotype in androgen receptor-positive prostate cancer [20]. Mancini et al. demonstrated that knockout of GABPB1L diminishes GABPA accumulation leading to reduced TERT expression, telomere loss, eventual apoptosis, and loss of tumorigenic potentials in TERT promoter-mutated glioblastoma cells [26]. These findings supported GABPA as a cancer driver. It is currently unclear why and how this happens and what the detailed mechanism is. One of potential explanations is that GABPA is a transcription factor and may regulate various downstream genes, so, how GABPA works may depend on different cell contexts and tumor types. In immunohistochemistry studies, we also found that the GABPA protein expressed in cell cytoplasm as well as in the nucleus. Exact mechanism of GABPA in EC remains further studies to elucidate. Besides serving as a transcription factor, we speculated that GABPA may play its role through other approaches.

Most EC patients can be cured with surgery only, but patients at advanced-stage or some early-stage patients will recur. Therefore, it is vital to identify novel biomarkers to detect EC recurrence and predict the prognosis. In our study, we demonstrated that the expression of GABPA corelated with patients' prognosis. We also found that the expression of GABPA in EC is related to some clinicopathological features, including pathologic types and histologic grade based on TCGA. The Kaplan-Meier analysis and log-rank test suggested that patients with a lower level of GAPBA had worse OS and DFS. Univariate and multivariate Cox regression analyses revealed that the downregulation of GABPA is related to poor prognosis in EC. We provided convincing evidence that GABPA can act as an independent predictor of EC. Our study agrees with several recent investigations, which showed that the lower GABPA expression is correlated with bigger tumor sizes, advanced stages or grades, local and distant metastasis, and poor outcomes in patients with thyroid carcinoma, hepatocellular carcinoma, or bladder cancer [17, 18, 22]. Also, lower expression of GABPA is associated with shorter 5-year survival in clear cell renal cell carcinoma and colorectal and head neck cancer based on TCGA database [24].

Therefore, the present study points out that GABPA may act as a tumor suppressor, and it could be considered as a potential prognostic biomarker for EC.

## 5. Conclusion

In summary, our study showed that GABPA was downregulated in EC tissues which may be associated with its methylation. The low GABPA expression was associated with some clinicopathological characteristics and poor survival in EC patients. Our research indicates that GABPA may serve as a potential marker for EC and be useful for the treatments against EC.

## Figures and Tables

**Figure 1:** The expression of GABPA in EC patients was analyzed by TCGA database. (a) The transcript level of GABPA in EC tissues and normal endometrial tissues. (b) The expression of GABPA in 23 paired samples (EC tissues and its adjacent normal tissues). (c) The expression of GABPA in different pathological types of EC. (d) The expression of GABPA in two types of EC. (e) The expression of GABPA in different grades of EC. (f) The expression of GABPA in different stages of EC.

**Figure 2:** Kaplan-Meier survival analysis of the GABPA expression in EC patients by the TCGA database. (a) Effect of the GABPA expression on overall survival in EC patients. (b) Effect of the GABPA expression on disease-free survival in EC patients.

**Figure 3:** Subgroup analyses of the GABPA expression in EC patients by the TCGA database. (a) Effect of the GABPA expression on overall survival in type II EC patients. (b) Effect of the GABPA expression on disease-free survival in type II EC patients. (c) Effect of the GABPA expression on overall survival in grades 3 EC patients. (d) Effect of the GABPA expression on disease-free survival in grades 3 EC patients.

**Figure 4:** Representative immunohistochemistry staining of GABPA in EC tissues. (a) Blank control staining. (b) Weak intensity. (c) Moderate intensity. (d) Strong intensity.

**Figure 5:** The expression of GABPA in EC patients was analyzed by IHC. (a) The expression of GABPA in normal tissues. (b) The expression of GABPA in EC tissues. (c) The protein level of GABPA in EC tissues and normal tissues.

**Figure 6:** Kaplan-Meier survival analysis of the GABPA expression in EC patients by IHC. (a) Effect of the GABPA expression on overall survival in EC patients. (b) Effect of the GABPA expression on disease-free survival in EC patients.

**Figure 7:** The association of GABPA mRNA and its gene methylation was analyzed by TCGA database. (a) The association between the GABPA mRNA expression and its gene methylation. (b) The association between the GABPA mRNA expression and methylated CpG of cg21890848 at the GABPA gene.

**Table 1:** Clinicopathologic characteristics.

Characteristic	*N*	(%)
Age (year)	63.70 ± 11.87	
Histology		
Endometrioid	377	76.94
Serous	92	18.78
Mixed serous and endometrioid	21	4.28
Grade		
G1	91	18.57
G2	114	23.27
G3	285	58.16
Stage		
I	308	62.86
II	50	10.20
III	109	22.25
IV	23	4.69
Surgical approach		
Open	279	56.94
Minimally invasive	189	38.57
No data	22	4.49
Peritoneal cytology		
Negative	325	66.33
Positive	47	9.59
No data	118	24.08
Adjuvant therapy		
Yes	299	61.02
No	191	38.98
GABPA expression		
Low	245	50.00
High	245	50.00

Age: age of endometria carcinoma diagnosis; GABPA: GA-binding protein A.

**Table 2:** Univariate and multivariate Cox regression analysis of the GABPA expression and overall survival in EC patients.

Variable	Univariable		Multivariable	
	HR (95% CI)	*P* value	HR (95% CI)	*P* value
Age (<60 vs ≥60)	1.747 (0.827-3.692)	0.144	—	0.215
Histology (type I vs type II)	2.237 (1.152-4.343)	**0.017** ^∗^	—	0.411
Grade (G1-2 vs G3)	2.933 (1.344-6.401)	**0.007** ^∗^	2.381 (1.068-5.310)	**0.034** ^∗^
Stage (stage I vs stage II-IV))	3.387 (1.935-7.607)	**≤0.001** ^∗^	3.033 (1.505-6.123)	**0.002** ^∗^
Surgical (open vs mini-invasive)	0.671 (0.313-1.436)	0.304		
GABPA (low vs high)	0.487 (0.246-0.966)	**0.040** ^∗^	0.491 (0.246-0.977)	**0.043** ^∗^

GABPA: GA-binding protein A; EC: endometrial carcinoma; age: age of endometria carcinoma diagnosis; HR: hazard ratio; CI: confidence interval; bold type and (^∗^) indicate statistical significance.

**Table 3:** Univariate and multivariate Cox regression analysis of the GABPA expression and disease-free survival in EC patients.

Variable	Univariable		Multivariable	
	HR (95% CI)	*P* value	HR (95% CI)	*P* value
Age (<60 vs ≥60)	1.680 (1.017-2.777)	**0.043** ^∗^	1.670 (1.011-2.760)	**0.045** ^∗^
Histology (type I *vs* type II)	1.629 (1.024-2.593)	**0.039** ^∗^	—	0.416
Grade (G1-2 vs G3)	1.499 (0.952-2.630)	0.081	—	0.332
Stage (stage I vs stage II-IV))	2.281 (1.482-3.511)	**≤0.001** ^∗^	2.219 (1.441-3.418)	**≤0.001** ^∗^
Surgical (open vs mini-invasive)	1.039 (0.657-1.643)	0.870		
GABPA (low vs high)	0.584 (0.375-0.910)	**0.018** ^∗^	0.619 (0.397-0.966)	**0.045** ^∗^

GABPA: GA-binding protein A; EC: endometrial carcinoma; age: age of endometria carcinoma diagnosis; HR: hazard ratio; CI: confidence interval; bold type and (^∗^) indicate statistical significance.

**Table 4:** Clinicopathologic characteristics.

Characteristic	*N*	(%)
Age(year)	55.16 ± 9.74		
Histology			
Endometrioid	88	82.24	
Serous	13	12.15	
Mixed serous and endometrioid	6	5.61	
Myometrial invasion			
<50%	71	66.36	
≥50%	36	33.64	
Cervical invasion			
Negative	97	90.65	
Positive	10	9.35	
Lymph nodes			
Negative	92	85.98	
Positive	15	14.02	
Grade			
G1	47	43.93	
G2	36	33.64	
G3	24	22.43	
Stage			
I	85	79.44	
II	3	2.80	
III	18	16.82	
IV	1	0.94	
Surgical approach			
Open	98	91.60	
Minimally invasive	9	8.40	
GABPA expression			
Low	64	59.81	
High	43	40.19	

Age: age of endometria carcinoma diagnosis; GABPA: GA-binding protein A.

**Table 5:** Univariate and multivariate Cox regression analysis of the GABPA expression and overall survival in EC patients.

Variable	Univariable		Multivariable	
	HR (95% CI)	*P* value	HR (95% CI)	*P* value
Age (<60 vs ≥60)	1.810 (0.730-4.491)	0.200		
Histology (type I vs type II)	2.007 (0.634-6.357)	0.236		
Grade (G1-2 vs G3)	2.538 (0.933-6.901)	0.068	—	0.587
Stage (stage I vs stage II-IV))	2.099 (1.321-3.334)	**0.002** ^∗^	3.725 (1.475-9.407)	**0.005** ^∗^
GABPA (low vs high)	0.257 (0.075-0.881)	**0.031** ^∗^	0.267 (0.078-0.918)	**0.036** ^∗^

GABPA: GA-binding protein A; EC: endometrial carcinoma; HR: hazard ratio; CI: confidence interval; age: age of endometria carcinoma diagnosis. Bold type and (^∗^) indicate statistical significance.

## Data Availability

The data used to support the findings of this study are available from the corresponding author upon request.
